# PD-L1 rs2890658 Polymorphism Increases Risk for Non-Small-Cell Lung Cancer in Northern China Population Based on Experimental Data and Meta-Analysis

**DOI:** 10.1155/2022/8433489

**Published:** 2022-08-01

**Authors:** Guigang Wang, Yuehua Dong, Yanjun Yang, Wenjing Zhang, Na Liu, Yulei Wei

**Affiliations:** Thoracic Cardiovascular Surgery, The First Affiliated Hospital of Hebei North University, Zhangjiankou, Hebei, China

## Abstract

**Purpose:**

To dig the PD-L1 rs2890658 polymorphism with susceptibility of non-small-cell lung cancer (NSCLC) in northern China.

**Patients and Methods:**

There were 600 NSCLC patients and 600 age and sex matched controls from the same ethnic origin recruited in the present research. Polymerase chain reaction-restriction fragment length polymorphism method genotyped PD-L1 rs2890658 polymorphism. PubMed and Embase were searched to get eligible literature for meta-analysis. The association between PD-L1 rs2890658 polymorphism and NSCLC risk was calculated with odds ratio and 95% confidence interval.

**Results:**

It is more likely that individuals who have CC genotype and C allele are 2.15 and 1.41 times to develop NSCLC compared with individuals with AA genotype and A allele, respectively. Meta-analysis showed that the individuals who have C allele and CA genotype increased the risk of suffering from NSCLC.

**Conclusion:**

PD-L1 rs2890658 polymorphism increased NSCLC risk in northern China population and it might predict the occurrence of NSCLC.

## 1. Introduction

A large number of studies have shown that smoking is closely related to the incidence of lung cancer, and the risk of lung cancer among smokers is nearly 10 times higher than that of nonsmokers. In addition, China currently has more than 33% of the world's smokers [1]. Since the change in lung cancer incidence lags behind the smoking rate by about 20–30 years, the proportion of lung cancer incidence and death will be more prominent in the world in the near future. It can be seen that lung cancer has become one of the most important diseases threatening the whole world and people's lives and health in China, and it is a major public health problem that needs to be solved. As the main cause of cancer death across the world, lung cancer is divided into non-small-cell lung cancer and small-cell lung cancer, and NSCLC occupies about 85% of lung cancer. The onset of lung cancer is insidious. About 55% of patients with lung cancer suffer from metastasis during the first diagnosis, with a poor prognosis. The 5-year survival rate is 18%, while patients with advanced stages show a 5-year survival rate of only 5.5% [2, 3]. For a long term, patients with advanced lung cancer have received platinum-based chemotherapy as the standard first-line treatment, with large side effects and poor tolerance and an effective rate of only 25–35%, indicating to some extent that the efficacy of cytotoxic chemotherapy drugs has reached a platform. With the in-depth understanding of tumor signal transduction and pathways, the usage of targeted therapy gives novel hope to patients with lung adenocarcinoma, and the median survival time of patients with positive sensitive mutations after receiving targeted drugs is longer than that of patients without sensitive mutations. However, patients with sensitive mutation-negative nonsquamous non-small-cell lung cancer and lung squamous cell carcinoma cannot benefit from targeted therapy. In this case, the emergence of immunotherapy has changed the existing treatment strategy of NSCLC, and immune checkpoint inhibitors have made great achievements in the clinical application of NSCLC.

Immune checkpoint inhibitors physiologically control the immune response by blocking inhibitory pathways, restoring and maintaining the immune system against cancer cells. As the earliest clinically developed receptor targeting immune checkpoints, CTLA-4 [4] is mainly shown on activated T cells and regulatory T cells and controls the immune response at the early stage of T cell activation by inhibiting helper T cells and enhancing the activity of regulatory T cells [5]. Recently, programmed cell death ligand-1 has been a hot gene in tumor immunotherapy and a potential molecular target for predicting drug efficacy [6]. The PD-L1 protein encoded by this gene is widely expressed in a variety of solid tumor cells [7, 8]. When PD-L1 of tumor cells binds to PD1 on the T cell surface, it leads to proliferation inhibition, apoptosis, and inactivation of T cells, leading to immune escape of tumor [9]. Previous study has shown that PD-L1 overexpression is a predictor of poor prognosis [10]. It was found that single nucleotide polymorphism of PD-L1 gene can regulate the expression of PD-L1 protein in gastric cancer and lung cancer and affect the prognosis of patients [11, 12]. Besides, PD-L1 polymorphism is also related to the risk of liver cancer [13], gastric cancer [14] and lung cancer [15]. However, the relationship between PD-L1 polymorphism and NSCLC susceptibility is still unclear. Several gene polymorphisms of the PD-L1 gene have been detected in Asian population, where the rs2890658 polymorphism (8923 A/C) has been widely investigated and reported. This SNP can be detected in the Chinese population and is linked with multiple diseases [16–19]. Nevertheless, literature about this polymorphism in NSCLC is rare and has inconsistent results. Therefore, we evaluate the PD-L1 rs2890658 polymorphism with NSCLC susceptibility with a large sample size to derive a more accurate result.

## 2. Materials and Methods

### 2.1. Research Object

There were 600 registered patients in Hebei who were diagnosed with NSCLC in the First Affiliated Hospital of Hebei North University from 2011 to 2021 in the case group. According to the classification standard of lung cancer tissue type of the WHO, the case group was divided into squamous cell carcinoma or adenocarcinoma by pathological type. In addition, the international lung cancer clinical staging system was used for clinical staging, and the case group was divided into stages I, II, III, and IV. The inclusion criteria for the case group are as follows: (a) newly diagnosed lung cancer cases with registered residence in Hebei province; (b) the patients who had not received antitumor therapy such as radiotherapy or chemotherapy; (c) the patients who had not suffered from other malignant tumors or other systemic diseases. There were 600 healthy subjects who received physical examination in the First Affiliated Hospital of Hebei North University in the control group. The inclusion criteria for the control group are as follows: (a) individuals with registered residence in Hebei Province; (b) they had no lung space occupying lesions, no irritating dry cough, bloody sputum, chest pain, or other malignant tumors. All subjects were unrelated Han individuals. The Ethics Committee of the First Affiliated Hospital of Hebei North University agreed the research protocol and experimental method of the current research, and all the individuals participating in this study have known and signed informed consent.

### 2.2. Sampling Collection, Genomic DNA Extraction, and Genotyping Analysis

The collection of a 5 mL venous blood sample was made by applying ethylenediamine tetraacetic acid (ethylenediaminetetraacetic acid, EDTA) or heparin anticoagulation. Using a whole blood genomic DNA extraction Kit, DNA was extracted. The concentration and purity of DNA were measured by an ultrafine uV-vis spectrophotometer. Polymorphism was genotyped by the PCR-RFLP technique. The PCR reaction process was as follows: predenaturation at 94°C for 3 min, denaturation at 9, denaturation at 94°C for 15 s, annealing at 55°C for 15 s, and extension at 72°C for 30 s, with a total of 35 cycles. Finally, it was extended for 3 min at 72°C. PCR amplified products were digested by enzyme and agarose gel electrophoresis was performed to observe the band position of the digested product and determine the genotype. The primer sequences product sizes for PD-L1 rs2890658 polymorphism were as follows according to the literature [20]: Forward: 5′-AATGGCTTGTTGTCCAGAGATG-3′; reverse: 5′-GTACCACATGGAGTGGCTGC-3′.

### 2.3. Data Collection

Two authors independently searched Pubmed and EMBASE. Search time starts on a database basis and ends in December 2021. And the keywords were shown below: “polymorphism” or “polymorphisms,” “non-small-cell lung cancer” or “NSCLC,” “PD-L1” or “programmed cell death ligand-1.” Only English and Chinese language studies were recruited. Furthermore, for no negligence of related literature, the references were searched.

### 2.4. Inclusion and Exclusion Criteria

The inclusion standards are as follows: (a) a case-control research evaluating the relationship between PD-L1 rs2890658 polymorphism and NSCLC risk; (b) enough data to count OR and 95% CI. The exclusion standards are shown below: (a) not a case-control research; (b) no adequate information to count OR and 95%CI. (c) experiment object of animals.

### 2.5. Data Extraction and Methodological Quality Assessment

The first author and second author strictly searched and evaluated all the data and information based on inclusion and exclusion criteria. Literature name, control source, genotyping methods, Newcastle-Ottawa Scale mark and HWE are necessary elements. In the case of different opinions between the first and second authors, the corresponding author will take part in the exploration and determination of the final outcomes. A similar approach was equally adopted to evaluate literature quality. The current meta-analysis evaluated the quality of each literature with the risk evaluation criteria of Newcastle-Ottawa Scale (NOS) bias. The major criteria were made up of three aspects, namely, selecting enrolled research subjects (0–4 marks); between-group comparability (0–2 marks); and exposure results and elements (0–3 marks). In addition, the ethics review and patient agreement were waived because neither human beings nor animals were involved.

### 2.6. Statistical Analysis

This relationship's power was evaluated with both the OR and 95%CI. The heterogeneity degree was evaluated with the *Q*-statistic and *I*^2^ statistics. There were four genetic models adopted to evaluate the relationship between PD-L1 rs2890658 polymorphism and NSCLC risk as the past literature reported. The fixed-effects or random-effects model was selected on the basis of the heterogeneity degree. It was considered that *I*^2^ < 50% is low heterogeneity, 50 ≤*I*^2^ < 75% is moderate heterogeneity, and *I*^2^ ≥ 75% is great heterogeneity. If *I*^2^ < 50% and *P* > 0.1, the fixed-effects model would be adopted. If *I*^2^ ≥ 50% or *P* ≤ 0.1, the random-effects model would be adopted. Sensitive analysis and publication bias were according to past meta-analysis. The current meta-analysis was made and disclosed according to the Preferred Reporting Items for Systematic Reviews and Meta-Analyses 2009 checklist [21]. SPSS 18.0 was responsible for all statistical analysis, including *t* test, *χ*^2^ test. The association between risk factors and ovarian cancer was evaluated by counting OR together with 95%CI and performing binary logistic regression. *P* < 0.05 was considered as great diversity.

## 3. Results

### 3.1. General Information of Study Subjects

Table 1 showed the detailed information of experimental group and control group. No great diversity was observed between NSCLC group and control group including gender, age, smoking history, or family history of cancer (*P* > 0.05).

### 3.2. Genotyping and Allele Distribution of PD-L1 rs2890658 Polymorphism

The PCR-RFLP method detected three kinds of genotypes (AA, AC, and CC) in both the NSCLC group and the control group. Significant associations were found between the NSCLC group and the control group for genotype and allele comparison. Individuals who have the CC genotype are 2.15 times more likely to develop NSCLC individuals than who have the AA genotype. Similarly, individuals who have the C allele are 1.41 times more likely to develop NSCLC than individuals who have the A allele. The detailed information is shown in Table 2.

### 3.3. Study Characteristics

The PRISMA 2009 flow diagram displayed the flow diagram of the current meta-analysis search process (Figure 1). Four Chinese literature were included in the meta-analysis altogether [22–25]. Major data of all literature are listed in Table 3. The genotyping methods were used only by PCR-RFLP. The publication year varied from 2012 to 2020, and all the controls were based on population. All the genotyping frequencies of controls were consistent with HWE. And the sample scale varied from 532 to 1128. The outcomes of NOS displayed the quality of all research and the mean mark was 8.2 according to Table 4.

### 3.4. Allele and Genotype-Wide Meta-Analysis

Thepositive outcomes between PD-L1 rs2890658 polymorphism and NSCLC risk by allele contrast (OR: 1.53, 95%CI=1.09-2.13, *P* = 0.013) is shown in Figure 2, heterozygous comparison (OR: 1.50, 95%CI = 1.04–2.16, *P* = 0.030) is shown in Figure 3, and dominate genetic model (OR: 1.54, 95%CI = 1.07–2.21, *P* = 0.019) is shown in Figure 4. Major outcomes between PD-L1 rs2890658 polymorphism and NSCLC risk are according to Table 5.

### 3.5. Evaluation of Between-Study Heterogeneity

Of the overall population, there was moderate heterogeneity under four genetic models (67.4%, 61.5%, 34.3%, and 71.8%). Therefore, we conduct subgroup analysis based on ethnicity to detect the heterogeneity source. Consequently, ethnicity was the main source of heterogeneity as the I^2^ of four genetic models of the Caucasian population was <50%(0, 0, 0, and 33.8%, respectively) after subgroup analysis was performed. If we eliminated the study from India, the degree of heterogeneity obviously reduced as almost no heterogeneity was found in the Brazilian or Caucasian population (Table 2).

### 3.6. Sensitivity Analysis and Publication Bias

Regardless of the literature excluded, the outcome of our meta-discussion was the same, suggesting the conformance and steadiness of the current meta-discussion. The outcome of sensitive discussion displayed stable present outcomes. No significant asymmetry was observed by funnel plot, and Egger's test also indicated that there was no significant asymmetry (*P* = 0.560).

## 4. Discussion

Immune checkpoint inhibitors have achieved good efficacy in the treatment of various tumors [26–30]. Its mechanism of action is to specifically stop PD-1 on the surface of T cells or the ligand PD-L1, avoiding tumor immune escape and enhancing the antitumor effect of the autoimmune system. These drugs are also effective for lung cancer, especially for those insensitive patients with chemotherapy and targeted therapy. Since the US FDA approved the first immune checkpoint inhibitor, Durvalumab, in 2018 for use in patients with stage III NSCLC, immunotherapy has been included in the 2019 NCCN lung cancer treatment guidelines and has been continuously updated. The suitable population characteristics of immune checkpoint inhibitors are different, which can bring more lasting survival benefits to suitable patients. Adverse reactions are also different from those of previous chemotherapy and targeted therapy. Patients have a good tolerance to immunotherapy, and most adverse events are controllable, while a few may lead to serious consequences. The side effects are mostly immune-related, such as immune pneumonia, myocarditis, enteritis, abnormal liver and kidney function, rash, hyperthyroidism, hypothyroidism, and type 1 diabetes.

Immunotherapy has become an emerging cancer treatment method in recent years. Different from traditional chemotherapy, immunotherapy enhances or normalizes the antitumor immune response by using the body's immune system so as to inhibit and kill tumor cells. Immunotherapy, shown by PD-1/PD-L1 checkpoint inhibitors, is one of the most potential study directions in the field of cancer therapy. It offers long-lasting benefits and is gradually becoming a first-line treatment in the guidelines. However, current studies suggest that not all populations benefit from pD-1/PD-L1 checkpoint inhibitors, especially first-line therapy in patients with advanced NSCLC. Therefore, it has become a hot topic to find an optimal detection index to screen the best beneficiaries. Many existing researches have displayed that the different expression levels of PD-L1 have a certain impact on the efficacy. With the accumulation of more and more clinical data, PD-L1 has become a relatively effective detection index at present, but its critical value is still controversial, and it has not been decided whether to take various treatments for patients with different expression results of PD-L1. However, the association between PD-L1 polymorphism and NSCLC susceptibility is still unclear. Therefore, the present study has evaluated the PD-L1 rs2890658 polymorphism with NSCLC susceptibility based on experimental data and meta-analysis. The outcomes of the meta-analysis indicated that AC genotype and C allele increased NSCLC risk. Our experimental data indicated that CC genotype and C allele grew NSCLC risk. Although we are driving somewhat inconsistent results, it is a very normal phenomenon when conducting gene polymorphism association studies [31, 32]. China has a vast territory and a large population. China has a population of over 1.4 billion with 56 ethnic groups. Varied regions and ethnic groups may have different genetic polymorphisms. Therefore, in this context, it is necessary to carry out meta-analysis and original research with a large sample size. In addition, we must acknowledge that the present paper has some shortcomings or deficiencies which need to be improved in the future. Because of simple laboratory conditions and limited funds, we have to admit the fact that the sample size of the current study is small. In future studies, we will include more patients and healthy people to make our results more reliable.

With the continuous development of bioinformatics and medicine and the arrival of the era of big data, people are no longer satisfied with research at the level of tissue cells but have begun to shift to research at the level of molecular medicine [33–35]. This has greatly promoted the mutual development between bioinformatics and medicine. The occurrence and development of a disease is a complex biological process involving multiple genes. If the treatment is only based on the clinical characteristics such as pathological type, clinical stage, patient age, and gender in traditional medicine, the expected effect may not be achieved [36, 37]. At this point, bioinformatics techniques can be used to study the therapeutic mechanism at the molecular level. Therefore, we would like to combine bioinformatics techniques with the diagnosis, treatment, and prognosis of NSCLC.

## 5. Conclusion

PD-L1 rs2890658 polymorphism increased NSCLC risk in northern China population and it might predict the occurrence of NSCLC.

## Figures and Tables

**Figure 1:** PRISMA 2009 flow diagram.

**Figure 2:** Forest plot for the associations between PD-L1 rs2890658 polymorphism and NSCLC risk in northern China population through allele contrast (C vs. A. NSCLC, non-small-cell lung cancer; OR, odds ratio; CI, confidence interval.

**Figure 3:** Forest plot for the associations between PD-L1 rs2890658 polymorphism and NSCLC risk in northern China population through heterozygote comparison (AC vs. AA). NSCLC, non-small-cell lung cancer; OR, odds ratio; CI, confidence interval.

**Figure 4:** Forest plot for the associations between PD-L1 rs2890658 polymorphism and NSCLC risk in northern China population through dominate genetic model (CC/AC vs. AA). NSCLC, non-small-cell lung cancer; OR, odds ratio; CI, confidence interval.

**Table 1:** The participates characteristics of both NSCLC and control group.

Basic information		Control (*N* = 600)	NSCLC (*N* = 600)	*P*

Age		61.3 ± 10.0	62.5 ± 9.9	0.115

Gender				0.131
	Male	320	346	
	Female	280	254	

Smoking status				0.343
	Ever	224	240	
	Never	376	360	

Family history of cancer				0.330
	Yes	102	115	
	No	498	485	

Clinicopathological type				—
	I	—	130	
	II	—	147	
	III	—	95	
	IV	—	170	

Histology types		—		
	Squamous carcinoma	—	229	—
	Adenocarcinoma	—	371	

NSCLC, non-small-cell lung cancer.

**Table 2:** Genotype and allele frequencies of PD-L1 rs2890658 polymorphism in NSCLC and control population.

SNPs	Genotypes	Case (*n* = 600)	Controls (*n* = 600)	OR (95%CI)	*P*

PD-L1 rs2890658					

Codominant model	AA	177 (29.5)	197 (32.8)	1.00^ref^	
	AC	255 (42.5)	316 (52.7)	0.90 (0.69–1.17)	0.421
	CC	168 (28.0)	87 (14.5)	2.15 (1.55–2.99)	<0.001

Allele	A	609 (50.8)	710 (59.2)	1.00^ref^	
	C	591 (49.2)	490 (40.8)	1.41 (1.20–1.65)	<0.001

PD-L1, programmed cell death ligand-1; NSCLC, non-small-cell lung cancer.

**Table 3:** Main characteristics of all case-control studies included in meta-analysis.

Literature	Ethnics (Country)	Genotyping methods	Source of control	Sample size	HWE conformity	NOS

Chen et al.	Asian (China)	PCR-RFLP	PB	293/293	Yes	8
Ma et al.	Asian (China)	PCR-RFLP	PB	528/600	Yes	9
Cheng et al.	Asian (China)	PCR-RFLP	PB	288/300	Yes	8
Zhao et al.	Asian (China)	PCR-RFLP	PB	281/251	Yes	8

PB, population-based; HWE: Hardy–Weinberg equilibrium; RFLP, restricted fragment length polymorphism; NOS, Newcastle-Ottawa score.

**Table 4:** Quality assessment of the four case–control studies according to the Newcastle-Ottawa scale.

Literature	Selection of enrolled study subjects	Between-group comparability	Exposure outcomes and factors	Total

Moura et al.	2	3	3	8
Loganathan et al.	3	3	3	9
Wu et al.	2	3	3	8
Tseng et al.	2	3	3	8
Average	2.3	3.0	3.0	8.3

**Table 5:** Meta-analysis of the PD-L1 rs2890658 polymorphism and non-small-cell lung cancer risk.

Comparison	*N*	Test of association			Mode	Test of heterogeneity		
		OR	95%CI	*P*		*χ* ^2^	*P*	*I* ^2^

C versus. A	4	1.53	1.09–2.13	0.013	Random	9.86	0.020	69.6
CC versus. AA	4	1.75	0.92–3.33	0.089	Fixed	1.60	0.659	0
CA versus. AA	4	1.50	1.04–2.16	0.030	Random	9.34	0.025	67.9
CC versus. CA/AA	4	1.71	0.90–3.25	0.102	Random	1.27	0.735	0
CC/CA versus. AA	4	1.54	1.07–2.21	0.019	Random	9.66	0.022	69.0

OR, odds ratio; CI, confidence interval.

## Data Availability

All data generated or analyzed during this study are included in this published article.
